The article "Progress Report on Interventional Treatment for Bronchopleural Fistula" was published in 2023. Journal: Emerg Med Int.

# Progress Report on Interventional Treatment for Bronchopleural Fistula

**DOI:** 10.1155/2023/8615055

**Published:** 2023-06-22

**Authors:** Pei Zhao

**Affiliations:** The Second Hospital of Shanxi Medical University, Taiyuan 030001, Shanxi, China

## Abstract

**Objectives:**

Bronchopleural fistula (BPF) is a serious and life-threatening complication. Following the advent of interventional radiology, subsequent treatment methods for BPF have gradually diversified. Therefore, this article provides an overview of the present scenario of interventional treatment and research advancements pertaining to BPF.

**Methods:**

Relevant published studies on the interventional treatment of BPF were identified from the PubMed, Sci-Hub, Google Scholar, CNKI, VIP, and Wanfang databases. The included studies better reflect the current status of and progress in interventional treatments for BPF with representativeness, reliability, and timeliness. Studies with similar and repetitive conclusions were excluded.

**Results:**

There are many different interventional treatments for BPF that can be applied in cases of BPF with different fistula diameters.

**Conclusion:**

The application of interventional procedures for bronchopleural fistula has proven to be safe, efficacious, and minimally invasive. However, the establishment of comprehensive, standardized treatment guidelines necessitates further pertinent research to attain consensus within the medical community. The evolution of novel technologies, tools, techniques, and materials specifically tailored to the interventional management of bronchopleural fistula is anticipated to be the focal point of forthcoming investigations. These advancements present promising prospects for seamless translation into clinical practice and application, thereby potentially revolutionizing patient care in this field.

## 1. Introduction

Bronchopleural fistula (BPF) refers to a pathological communication between the trachea, bronchi, and pleural cavity, representing a rare but life-threatening complication, commonly triggered by lung surgery. This condition has an incidence rate of 1.9%, with mortality rates ranging from 18% to 50% [1]. BPF can be classified into central and peripheral types; central BPF involves the fistula junction between the pleura and the primary or segmental bronchi, whereas peripheral BPF is characterized by the fistula junction between the pleura and subsegmental bronchi or distal airways of the lung parenchyma [2]. Varoli et al. [3] described the time of onset following surgical intervention to classify fistulas as early (1 to 7 days), intermediate (8 to 30 days), or late (more than 30 days). Several factors can precipitate BPF, such as anemia, malnutrition, hypoproteinemia, early recurrence of malignant tumors, prolonged preoperative use of glucocorticoids, the presence of chronic obstructive pulmonary disease, respiratory dysfunction, lung infection, preoperative respiratory failure, long-term mechanical ventilation, bronchial artery damage due to excessive intraoperative free bronchi, excessive lymph node dissection, and prolonged postoperative ventilator assistance [4]. Typical clinical symptoms of BPF include a productive cough often seen in pleural effusions, subcutaneous emphysema, fever in the early stages (with body temperatures between 38-39°C), sudden dyspnea, lowered oxygen saturation and blood pressure, mediastinal emphysema, and potentially life-threatening tension pneumothorax [5]. The primary treatment approach for BPF is individualized and aimed at closing the fistula and eliminating the pus cavity [6]. There is a wide range of interventional, surgical, and conservative treatments for bronchopleural fistula (BPF). Interventional therapy methods mainly include sclerosing agents, plugging agents, laser therapy, cryotherapy, chemicals, biomaterials, tracheal stents, and occlusive devices. As a new technology, interventional therapy provides a crucial role in the clinical treatment of BPF due to its characteristics of light trauma, low cost, excellent effect, and minor adverse reactions. This article reviews the advancements in interventional therapies for BPF.

The article "Progress Report on Interventional Treatment for Bronchopleural Fistula" was published in 2023. Journal: Emerg Med Int.

## 2. Level of Evidence

The level of evidence included in this review was determined using the Centre for Evidence-Based Medicine (CEBM) grading system. Five levels of evidence have been specified. (1) Level 1 is a systematic review conducted after collecting all reliable data according to the specific treatment of a specific disease in a randomized controlled trial. (2) Level 2 is the result of a single randomized controlled trial with a sufficient sample size. (3) Level 3 is a study with a control group but without group randomization. (4) Level 4 is an uncontrolled series of case observations. (5) Level 5 is a diagnosis and treatment plan proposed based on years of personal clinical experience of experts. Evidence levels 1 and 2 are classified as “high-level evidence,” level 3 as “moderate level of evidence,” and levels 4 and 5 as “low-level evidence.”

## 3. Progress Report

### 3.1. Endobronchial Nasal Bronchial Lavage

The endobronchial nasal bronchial lavage (ENBL) procedure is a new, minimally invasive, and safe method particularly effective in treating bronchopleural fistulas postlobectomy with diameters exceeding 5 mm. The duration of the ENBL surgery is typically between 10 and 15 minutes. In a study by Ning et al. [7], 17 patients postlobectomy with bronchopleural fistulas were recruited. A bronchoscope was employed to guide the ENBL tube from the nostril, through the trachea and bronchus, and into the pleural cavity via the fistula. The pleural cavity was then irrigated using the ENBL tube and subsequently drained via the thoracic drainage tube. Although patients reported minor adverse reactions including coughing, nausea, and sore throat, overall patient compliance was satisfactory with no instances of uncontrolled bleeding, pneumonia, or tracheal injury related to the procedure. Follow-ups were carried out for a minimum of six months postprocedure without requiring further intervention.

The article "Progress Report on Interventional Treatment for Bronchopleural Fistula" was published in 2023. Journal: Emerg Med Int.

### 3.2. Sclerosing Agents

Injecting sclerosing agents forms a local edema of the bronchial mucosa that surrounds the fistula and causes the fistula to become significantly smaller or even disappear, while the number of bubbles escaping from the thoracic drainage tube decreases substantially. As the edema decreases and the fistula reappears, the bubbles in the thoracic drainage tube will increase. Subsequently, the injection of sclerosing agents will lead to the development of submucosal inflammatory reactions and the intensification of local tissue proliferation, resulting in a reduction in the fistula. Generally, local tissue hyperplasia reaches its peak within a week. If the fistula has not yet closed, reinjecting the sclerosing agent into the surrounding submucosa is the key to a successful treatment [8].

#### 3.2.1. Aethoxysklerol

Aethoxysklerol is extensively used domestically and internationally, with few complications and excellent occlusion. Taking aethoxysklerol as the research object, a new drug, Lauromacrogol, which is composed of 1% aethoxysklerol, was studied and produced. In addition, Lauromacrogol, which is chemically known as polyoxyethylene lauryl ether, is a cleansing and sclerosing agent with surface activity. By altering the interface energy distribution, sclerotherapy can precipitate proteins in the cell within a few seconds, thereby damaging the cell membrane lipid bilayer and causing the cell membrane to rupture, alongside sterile inflammation, cell necrosis, fibrous tissue proliferation, and adhesions [9]. Fibrotic bronchoscopy-guided injection of 1% aethoxysklerol into the BPF can both safely and effectively close the fistula and also be injected repeatedly without affecting subsequent treatments. Most fistulas can be successfully closed with a single injection if the fistula diameter is less than 3 mm; however, for patients with fistula diameters greater than 3 mm, the number of injections around the fistula increases significantly. As long as the fistula diameter is less than 6 mm, the success rate of closure remains relatively high. This is consistent with the results reported by Ge et al. [8].

The article "Progress Report on Interventional Treatment for Bronchopleural Fistula" was published in 2023. Journal: Emerg Med Int.

#### 3.2.2. Ethanol

Absolute ethanol sclerotherapy is suitable for difficult and potentially destructive lesions to achieve minimally invasive treatment, which has the advantages of no scarring, a low recurrence rate, and fewer complications compared to traditional surgery [10]. Ethanol has a therapeutic effect on BPF by causing a local inflammatory response, which leads to rapid tissue dehydration and protein denaturation, followed by fibrotic scarring. Abramian et al. [11] reported that two patients with BPF were treated with targeted submucosal injections of ethanol using the Olympus No. 21 endobronchial ultrasound-guided transbronchial needle aspiration (EBUS-TBNA) which could be performed bedside and resulted in favorable outcomes. However, the disadvantages of this treatment include the need for the operator to possess a high level of bronchoscopy expertise; the risk of organismal damage, such as ischemia and necrosis; and catastrophic damage to adjacent main blood vessels caused by improper injection.

#### 3.2.3. Ethanolamine Oleate

Small (<1 cm) BPFs can be closed through endoscopic injection for ethanolamine oleate (EO) hardening after a limited number of treatment courses. Its irritating action is effective in inducing rapid dehydration and scarring of the tissue. In a prospective observational descriptive study [12], 6 out of 8 (75%) BPF patients who received endoscopic treatment with ethanolamine oleate (EO) presented complete fistula closure without fistula reopening or serious complications. The study suggests that EO may be an effective treatment option for specific patients. Rivo et al. [13] described their experience in treating postoperative bronchial fistulas using ethanolamine and lauryl alcohol 400 under bronchoscopy. Furthermore, only one of eight patients was unable to complete the treatment due to a pathological recurrence of the tumor, while the fistula persisted. In another 7 cases (87.5%), fistula closure was successful. This is similar to the research findings of Varoli et al. [3]. The submucosal injection of ethanolamine and lauryl alcohol 400 around the bronchoscopy fistula is a minimally invasive, effective, and safe method for the treatment of BPF. Controlling against infection before treatment, adequate drainage, multiple injections during treatment, and repeated injections either at one time or multiple times can help improve the success rate of the treatment [14].

### 3.3. Plugging Agents

The plugging agent can both directly plug the fistula and cause inflammation of the mucosa near the fistula to promote local tissue fibrosis and block the fistula. Therefore, plugging agents, such as fibrin glue, a synthetic hydrogel, polyvinyl alcohol (PVA) sponge, and cyanoacrylate glue, are used to treat airway fistulas.

The article "Progress Report on Interventional Treatment for Bronchopleural Fistula" was published in 2023. Journal: Emerg Med Int.

#### 3.3.1. Fibrin Glue

Fibrin glue, also called fibrin adhesive, is a biological product isolated from human plasma, while its main components are thrombin, fibrinogen, and other preparations. Fibrin glue has a myriad of functions, such as hemostasis, sealing and bonding wounds, and preventing tissue adhesion. The mechanism of action for fibrin glue simulates the final step of blood coagulation, i.e., when thrombin interacts with calcium ions, fibrinogen molecules cleave to produce fibrin peptides A and B, which leads to the formation of fibrin monomers. Simultaneously thrombin also activates factors that involve the cross-binding of fibrin and the formation of stable, nonfragile fibrin clots. Tang and Rong [15] used an OLYMPUS electronic bronchoscope to enter the bronchi and locate the fistula, then removed the fistula secretion, placed a thin catheter along the bronchoscopic biopsy tube into the fistula, and injected 2-3 mL of fibrin glue through the catheter under direct vision, which can form an instant polymer adhesive to close the fistula. Fibrin glue injection for BPF treatment has its advantages, including minimal trauma, few complications, and repetition. In addition, it is suitable for BPF with a fistula diameter of less than 5 mm, although cough suppressants need to be used after surgery to prevent the adhesion block from falling off due to the onset of an irritating cough.

#### 3.3.2. Hydrogel

Hydrogel is a three-dimensional network-structure material composed of macromolecules and water molecules. It has good biocompatibility, hemostasis, and tissue regeneration-promoting properties and is widely used in the field of biomedicine. The upregulation of phosphorylation levels of the signal transduction and transcriptional activator protein 3 can promote the polarization of megaphage cells to the anti-inflammatory M2 phenotype, reduce the inflammatory response of chronic wounds, and promote the transition from chronic wounds to the proliferation phase, ultimately, accelerating wound healing. Shahrouki et al. [16] reviewed five patients with BPF after lung ablation from 2009 to 2017. These patients were given a synthetic hydrogel sealant through the skin under the guidance of computed tomography (CT). Four patients had their air leakage at the fistula completely resolved without immediate complications, and there were no signs of delayed complications or recurrent air leakage during follow-up. They believed that the hydrogel was a potentially safe and effective alternative treatment for persistent air leakage at the fistula after lung ablation. Beckmann et al. [17] reported that 0.1 cc of carboxymethylcellulose (prolaryn gel) can be injected twice around the fistula to treat a newborn with laryngeal atresia and BPF, thus achieving significant results. The successful use of carboxymethylcellulose injection to treat BPF, by Beckmann et al., suggests that this procedure may help infants with persistent BPF to avoid segmental lung resection.

The article "Progress Report on Interventional Treatment for Bronchopleural Fistula" was published in 2023. Journal: Emerg Med Int.

#### 3.3.3. Rapid Medical Adhesive

The rapid medical adhesive has good tissue compatibility, is nontoxic, and can be gradually degraded and absorbed after completing its intended use. For example, medical OB adhesive is 1 of the 508 series of rapid medical adhesives, chemically known as *α*-cyanoacrylate, which is a liquid type of rapid medical adhesive. It can rapidly polymerize with the biological tissue at room temperature when it encounters blood on a person's wound surface or when the tissue fluid contains trace amounts of anionic substances or organic amines. After curing into a film in 15 seconds, the adhesive film is tightly embedded in the surface of the wound, enabling the tissue at the sutured incision or anastomotic opening to be firmly adhered and sealed, closing these wounds, stopping the bleeding, and separating the adhesive tissue from bacteria to create a wound protection effect. It also creates a good growth environment for lung tissue sections, bronchial stumps, or bronchoplasty, which benefits the early healing of the fistula. BPF with a fistula diameter of less than 5 mm can be sealed with glue under bronchoscopy, which can be repeatedly operated on with minimal adverse reactions and no serious complications. It can significantly improve the pressure resistance of the trachea. In a study by Lin et al. [18], iodophor, silver nitrate, and a medical adhesive (OB glue) were locally administered via fiberoptic bronchoscopy to five patients with bronchopleural fistulas of approximately 0.3–0.5 cm in diameter after pneumonectomy, with satisfactory results. The medical adhesive, being devoid of toxic side effects, readily solidifies into a film upon local application within the body. This process serves to protect the wound surface, strengthen tissue, promote healing, and facilitate absorption by the body. Iodophor acts as a potent bactericidal disinfectant, and a 0.2% silver nitrate solution exhibits astringent properties, sterilizes, and encourages the healing of ulcers and erosions. This therapeutic approach for chronic empyema and bronchopleural fistulas, delivered through fiberoptic bronchoscopy, has proven straightforward to implement and minimally painful for the patients. Battistoni et al. [19] performed endoscopic treatment on 7 patients with a fistula diameter of 4–8 mm. They used rigid bronchoscopy to insert the small cylinder of PVA sponge into the fistula and then directly coated the cyanoacrylate adhesive to the PVA sponge through the channel catheter, once a month for 3 months, to achieve good results. Thus, PVA sponges filled with liquid cyanoacrylate are considered an effective treatment method for chronic and large fistula patients and are suitable for different parts, shapes, and sizes of BPF. The local application of iodophor, silver nitrate, and OB glue, as performed by Lin Qing et al., has demonstrated promising outcomes in the treatment of bronchopleural fistulas of roughly 0.3–0.5 cm in diameter. However, it remains to be investigated whether this therapeutic approach exhibits therapeutic efficacy for patients with bronchopleural fistulas larger than 0.5 cm in diameter. Battistoni achieved therapeutic success in patients with bronchopleural fistulas greater than 0.5 cm in diameter using a combination of cyanoacrylate adhesive and PVA sponge. This indicates that this combined method might represent a feasible and effective treatment for bronchopleural fistulas of a diameter larger than 0.5 cm.

The article "Progress Report on Interventional Treatment for Bronchopleural Fistula" was published in 2023. Journal: Emerg Med Int.

### 3.4. Laser Therapy

For clinically small or cribriform fistulas, laser ablation of the mucosa adjacent to the fistula can induce tissue edema and protein degeneration, stimulate local inflammatory reactions, and achieve fistula healing in the form of tissue fibrosis. Using a laser to repair the fistula is a noninvasive, cost-effective, and effective new method for treating BPFs after lobectomy. This treatment is mainly applicable to patients with a fistula diameter of less than 2 mm and requires no obvious tumor involvement or infection signs in the bronchial stump. However, due to the frequent presence of local infections in the bronchial stumps, stubborn chest infections, or large amounts of pleural effusion in patients with BPF, the clinical application of laser therapy is limited.

### 3.5. Cryotherapy

Rapidly cooling and freezing diseased tissue can cause freezing necrosis, exudation, adhesion, and scar formation, which can quickly remove dead and damaged materials without disrupting normal mucosal growth. The fistula eventually heals by forming a firm scar from many collagen strands. Thus, setting the freezing temperature, time, and frequency correctly can yield good results without significant complications. Therefore, cryotherapy has the advantages of minimal trauma, low cost, and safety.

The article "Progress Report on Interventional Treatment for Bronchopleural Fistula" was published in 2023. Journal: Emerg Med Int.

### 3.6. Chemical Substances

The implementation of this method requires the injection volume to not be too large at once; otherwise, it may overflow, stimulate, and damage surrounding normal tissues. During the operation of fibrotic bronchoscopy, endotracheal surface anesthesia should be fully performed to ensure good patient cooperation. Due to local stimulation, it is likely to cause severe coughing, causing chemicals to enter the lobar and main bronchi and affect the mucosa in this area. Therefore, the fistula location should be accurately determined, and if necessary, methylene blue can be injected to determine the location of the BPF.

#### 3.6.1. 100% Carbolic Acid

Pure carbolic acid (100%) has low corrosivity to the mucosal tissue. When it comes into contact with the mucosal surface, the tissue quickly turns pale and degenerates, leading to pathological processes such as inflammation, exudation, and proliferation of the mucosa, thereby closing the fistula without coughing up blood or having breathing difficulties. A small amount of acid overflow can cause an irritating cough and damage to the surrounding normal mucosa. This technique presents several advantages, including ease of implementation, patient comfort, and the lack of requirement for hospitalization. It is particularly effective for patients with substantial BPF coupled with pronounced pleural effusion and sputum, as it rapidly alleviates symptoms and circumvents aspiration pneumonia. The precise position, size, and shape of the fistula can be effectively determined, thereby reducing the surgical risk, mortality rate, and cost of treating BPF. Wang et al. [20] assessed 12 patients with BPF after pneumonectomy and achieved significant efficacy by instilling 100% carbolic acid into the mucosal surface around the fistula. During bronchoscopy treatment, all 12 patients did not exhibit bleeding, severe dyspnea, or a decrease in SpO2. The efficacy of the instillation method is accurate and safe; thus, for patients with BPF and a fistula diameter of <7 mm, poor general condition, and the one who cannot tolerate surgery, using a carbolic acid solution is a suitable option. However, difficulties may arise in healing if the fistula size exceeds a certain threshold, potentially due to insufficient stimulation of healthy mucosa for tissue proliferation and regeneration [21].

#### 3.6.2. 3% Trichloroacetic Acid

After spraying trichloroacetic acid onto the mucosal surface, the mucosa quickly becomes pale and even necrotic. Subsequently, pathological processes such as inflammation, exudation, and mucosal proliferation occur, causing the fistula to close. Yu et al. [22] injected 0.5–1 mL of 3% trichloroacetic acid into the fistula through nasal fibrotic bronchoscopy in 18 BPF patients, and the fistulas of 12 patients were closed within one week. Furthermore, five cases were injected with the second needle, while one case was completely closed following the third needle. These data were significant and did not present any complications, such as dyspnea.

The article "Progress Report on Interventional Treatment for Bronchopleural Fistula" was published in 2023. Journal: Emerg Med Int.

### 3.7. Biological Materials

Mesenchymal stem cells can exist in the bone marrow, fat, blood, umbilical cord, and other tissues. Moreover, they can be transplanted into the airways to form a dense epithelial tissue. Bone marrow mesenchymal stem cells (BMSCs) are self-renewing pluripotent stem cells that exist in the human bone marrow. Previous studies have shown that BMSCs achieve their therapeutic goals mainly through cell differentiation, paracrine, and immune regulatory mechanisms. Local injection of BMSCs under an endoscope can promote the proliferation of fibroblasts and collagen fibers in the fistula, thereby closing it and achieving the required therapeutic purposes. Furthermore, BMSCs possess advantages that are unrelated to medical ethics—for example, convenient material collection, easy isolation and cultivation, low immunogenicity, and multiple transplantation methods. Moreover, this method avoids the limitations experienced by using general biomaterials, such as vascular coils and gelatin foam. However, BMSCs still have shortcomings in the treatment of BPF [23]. Firstly, this form of treatment is mostly in the experimental stage, while the medical reports in clinical applications are few, and there remains a lack of multicenter and long-term follow-up data. Thus, insufficient evidence exists to support the therapeutic efficacy and mechanism of BMSCs. In addition, the indications alongside the short-term and long-term side effects in the treatment of BPF with BMSCs are unknown.

#### 3.7.1. Autologous Adipose-Derived Stem Cells

Adipose-derived stem cells were first isolated from lipid aspirates and used without cell expansion. In addition, a BPF was detected through bronchoscopy, and the mucosa surrounding the fistula was ablated with an argon plasma coagulator. Then, the isolated stem cells were endoscopically injected into the de-epithelialized area and fistula. Bottoni et al. [24] have recently obtained success in endoscopic surgery using mesenchymal stem cell infusion to treat BPF. Autologous fat infusion (fat filling) was used to treat eight patients with BPFs larger than 8 mm in diameter, and recovery was noted for all cases. Díaz-Agero Álvarez et al. [25] successfully treated BPFs with autologous adipose-derived stromal cells in two patients under bronchoscopy. A 3-year follow-up showed that the fistula was successfully closed and maintained without treatment-related adverse reactions, nonlocal malignant recurrence, or improved quality of life. This indicates that using autologous adipose-derived stem cells under bronchoscopy is a feasible, safe, and effective method for BPF treatment. The use of autologous fat in the treatment of BPF presents multiple advantages, primarily its effectiveness. It proves beneficial not only in BPFs measuring less than 8 mm but also in those exceeding 8 mm in diameter. In addition, its tolerability is noteworthy. Given that autologous fat does not face rejection issues, patients can readily tolerate it [24].

The article "Progress Report on Interventional Treatment for Bronchopleural Fistula" was published in 2023. Journal: Emerg Med Int.

#### 3.7.2. Autologous Blood

Autologous blood is a safe and reliable adhesive material that is easy to obtain and has excellent histocompatibility. It can be used to avoid fever and a series of other adverse reactions caused by the introduction of allogeneic materials. Furthermore, autologous blood contains a large number of coagulation factors, fibrinogen, and fibronectin, which can promote adhesion between pleural ruptures. For example, hemocoagulase is a fast-acting hemostatic agent that can be used for local and intravenous hemostasis. It can promote the conversion of plasma-soluble fibrinogen to insoluble fibrin, coagulate wound blood, promote epithelial cell growth, and accelerate wound healing. In addition, thrombocytin is also contained in hemocoagulase to enhance the function of platelets [26]. Autologous blood combined with hemocoagulase provides a good blocking effect on microBPF. Chen and Gong [27] stopped 52 cases (77.61%) in 67 patients, whose pleural fistula was successfully located, by using autologous blood to block bubble escape without recurrence. In 11 patients (16.42%), the escape of air bubbles decreased and gradually stopped with no recurrence; thus, providing a total effective rate of 94.03%. Furthermore, during a 6-month follow-up, there was no recurrence. In addition, autologous blood occlusion is affordable, uses convenient materials, has a simple implementation, and has low adverse reactions, especially for elderly patients who find it difficult to tolerate general anesthesia and chest surgery. However, adverse reactions such as transient PaO_2_ reduction and mild fever may occur.

#### 3.7.3. Platelet-Rich Plasma

Platelet-rich plasma (PRP) is platelet plasma, which is obtained by centrifugation using different sedimentation coefficients of whole blood components, when the platelet concentration is 3–6 times higher than the basic level. It contains a variety of biologically active substances, such as cytokines, which promote tissue repair and regeneration [28]. Siddique et al. [29] reported a case of noncystic fibrobronchiectasis treated with PRP under bronchoscopy. A patient with a bronchial fistula after bilateral lung transplantation was treated with autologous PRP under bronchoscopy twice. The patient tolerated the operation, without any complications. A subsequent follow-up, a few weeks later, showed that the fistula was completely closed and healed. In addition, PRP is an autologous serum preparation that contains abundant platelets and is applied to tissues to release rich growth factors and enhance healing by increasing the production of collagen and fibroblasts.

The article "Progress Report on Interventional Treatment for Bronchopleural Fistula" was published in 2023. Journal: Emerg Med Int.

#### 3.7.4. Fistula Plug

Fistula plugs function as a framework for fibroblasts, fostering natural tissue growth, facilitating cellular proliferation and tissue healing, and aiding in the repair of damaged tissues. Sakata et al. [30] reported the use of flexible bronchoscopy to place FPs in 5 patients with BPF. Among them, 3 patients completely stopped air leakage within 4 days and 1 patient significantly reduced air leakage, thereby achieving success. Another patient experienced air leakage following implantation, which may have resulted from the FP implant integrating with the surrounding tissue. Therefore, FP implantation may also pose a displacement risk. However, Sakata posits that further technological modifications may improve BPF closure and success rates.

### 3.8. Tracheal Stents

There are many kinds of tracheal stents, including metal stents (Gianturco, Wallstent, and Ultraflex stents), nonmetallic stents (Dumon and Polyflex stents), hybrid stents (AERO and Dynamc stents), and biodegradable drug sustained-release stents. Currently, the clinical application of stents includes self-expanding metal stents and silicone stents. Stent occlusion, where the stent is placed in the lesion area with a stent release device to completely cover or close the orifice fistula, can be performed by monitoring with DSA. The stent can fully obstruct the fistula, effectively isolating the path between the airway and the infected pleural cavity. It halts the ingress of airway secretions, laden with a high bacterial count, into the pleural residual cavity, thus severing the infection source. Furthermore, it blocks the pathway from empyema to normal airways and lung tissue, inhibiting the overflow of substantial pleural residual pus into the airways and the consequent intrusion into normal lung tissue, thereby preventing persistent pneumonia. Tracheal stent placement is one of the main therapeutic methods for BPF intervention, although complications such as mucus blockage, irritating cough, migration, and intense foreign body sensation remain unavoidable challenges.

The article "Progress Report on Interventional Treatment for Bronchopleural Fistula" was published in 2023. Journal: Emerg Med Int.

#### 3.8.1. Fully Covered Self-Expandable Metallic Stent

A fully covered, self-expandable metallic stent is a safe, effective, and rapid minimally invasive treatment for tracheal fistula, especially for patients who cannot tolerate surgery or other treatment failures but have the possibility of stent removal and displacement. Cao et al. [31] retrospectively analyzed nine patients who underwent the placement of fully covered, self-expandable metal stents covering the tracheobronchial or bronchial from August 2005 to November 2011. Six patients were placed with L-shaped stents, and three patients were placed with I-shaped stents. The surgical time was 5–16 minutes. All patients successfully received the stents on the tracheobronchial tree without any surgery-related complications. One patient coughed out the stent 5 days after placement, 2 died of other complications, and 6 patients had empyema that subsided after 2 to 5 months (the recovery rate was 75%). A follow-up period of 3–36 months was implemented for seven patients. During the follow-up period, one stent was removed due to difficulty in expectoration eight months after placement, and there was no recurrent empyema. However, the rest of the patients had good stent tolerance, where it remained stable without migration or recurrence of empyema. For patients with left upper lobe bronchial fistula, an I-shaped stent is generally used; for right upper lobe bronchial fistula, an L-shaped stent should be used. For main bronchial fistulas and other cases, where stent placement was not appropriate in the affected airway, an L-shaped stent should be used instead [32]. Previous research suggests [33] that the I-shaped stent has a small contact area with the bronchial mucosa and a high displacement rate. The L-shaped blind end-covered stents and “Y”-shaped single bullet-covered stents can reduce the incidence of stent displacement by increasing the contact area between the stent and the tracheal mucosa. In addition, the L-shaped stent partially covering the tracheobronchial branches can effectively occlude the long stump BPF; the Y-shaped single warhead-covered stent has a good sealing effect on the BPF with short residual ends [34]. Li et al. [35] chose a customized Y-shaped self-expansive covered metal stent with dead corners, which was removed within 3 months to avoid granulation proliferation induced by long-term stent placement. In this case, the application of a Y-shaped, self-expanding, covered metal stent with a dead angle successfully occluded the fistula and promoted its healing. Airway stent placement is a relatively mature scheme for the interventional treatment of BPF. However, the increased contact area between the stent and the tracheal mucosa may affect the function of fibrous columnar epithelial cells in the airway mucosa and, in severe cases, may lead to sputum retention and lung infection. Therefore, it is recommended to conduct periodic chest multislice computed tomography (MSCT) scans to observe the closure of the fistula and the residual cavity size and to determine the appropriate timing for stent removal.

The article "Progress Report on Interventional Treatment for Bronchopleural Fistula" was published in 2023. Journal: Emerg Med Int.

#### 3.8.2. Silicone Stent

In 1987, French physician Dumon proposed and implemented silicone stents, which are now known as Dumon stents. They are available in straight cylindrical and Y-shaped structures, according to their appearance. Their clinical application began after entering the Chinese market in 2014. The use of a trimmed Y-shaped silicone stent can effectively solve the problem of airway stenosis, effectively block the fistula, eliminate air leakage in the airway, and significantly improve breathing difficulties [36]. Zeng et al. [37] retrospectively analyzed the records of 17 patients with BPF and found that in patients with modified Dumon stents placed under bronchoscopy, the air leakage stopped immediately in 16 patients (initial success rate: 94.1%). Only one patient failed to achieve initial success due to a failed match between the blocked branch and the airway. However, the stent placement was well tolerated. During the follow-up period, no airway rupture, asphyxia, laryngeal edema, or suture dehiscence occurred. Almost all patients reported coughing and poststernal pain after surgery; however, this was relieved by administering cough suppressants and analgesic regimens. Schweiger et al. used 3D printing technology to establish an in vitro model of a Y-type silicone airway stent to simulate the trachea [38], thereby completely solving problems such as patients having different trachea diameters, different angles between the central trachea and bronchus, and trachea length. Therefore, this technology achieved good compatibility between the stent and the patient's trachea.

### 3.9. Occlusive Devices

#### 3.9.1. Cardiac Occluders

Originally, the cardiac defect occluder was designed to treat congenital atrial ventricular septal defects and patent ductus arteriosus (PDA). In 2008, it was first reported that blocking BPF with an atrial septal defect (ASD) occluder could provide a significant clinical effect. With the development of interventional therapy technology and medical instruments, ASD occluders, ventricular septal defect (VSD) occluders, PDA occluders, and other occluders have been used to treat BPF. Therefore, some patients can achieve the goal of healing the fistula after treatment with occlusive devices, providing a new idea for BPF treatment [39].

*(1) ASD Occluder*. The main body of the atrial septal defect occluder is a double-disc structure connected through the waist. Thus, the ASD occluder uses the waist to provide support and seal the fistula. The bilateral discs play a certain role in isolating and fixing the occluder in the fistula, achieving effective occlusion through the coordination of the waist and the disc [40]. An atrial septal defect occluder can increase the coverage area of the fistula, improve the sealing effect, and reduce the incidence of occluder displacement. In their study, Fruchter et al. [41] utilized an ASD occluder to treat ten BPF patients. Success was noted in nine cases, while one patient experienced failure due to occluder dislodgement into the chest. Wang et al. [42] described two instances of BPF patients, both with fistula diameters of 6 mm, who initially showed limited response to multiple treatment modalities. Following treatment with an ASD occluder, both cases demonstrated improved outcomes and no recurrences during follow-up. Zhou et al. [43] applied the ASD occluder in a case of postoperative BPF in a lung cancer patient, with a fistula diameter of approximately 12 mm. Three months post-treatment, the patient's family reported no BPF recurrence and a stable lung condition. Ottevaere et al. [44] reported successful usage of an ASD occluder for a BPF with a 10 mm fistula diameter. Similarly, Papiashvilli et al. [45] used an ASD occluder in treating a BPF patient postpneumonectomy, who had a 4 mm fistula at the pneumonectomy stump corner and a 3 mm fistula in the right accessory bronchus area. Three years postoperatively, the patient maintained good overall health. These findings suggest that the ASD occluder can effectively serve in the interventional treatment of BPF patients with varying fistula sizes. ASD is mainly applicable to the treatment of bronchial stump fistulas in large airways (bronchi above grades 1–3). This occluder has good biocompatibility, promotes the growth of tracheal granulation tissue, and further enhances the occlusive effect. Furthermore, it is not necessary to remove the atrial septal defect occluder following implantation because it will not lead to an obstructed sputum excretion, although it may cause fistula dilation, fatal massive hemoptysis, nickel-titanium alloy wire breakage, and other occluder-related complications.

*(2) VSD Occluder*. The VSD occluder is a nitinol wire mesh woven into a double-disc structure, which forms a self-expanding implantable device. Bai et al. [46] used HeartR™ membrane ventricular septal defect occluders in 10 patients with postoperative BPF and closed the BPF by soft bronchoscopy under general anesthesia. During the follow-up period, the technical success rate was 100% and the complete closure rate was 70%; furthermore, there were no complications, and the physical tolerance was good. Notably, using a ventricular septal defect occluder to close BPF under bronchoscopy after pneumonectomy is considered a safe and effective method. Liu et al. [47] reported the successful implantation of a VSD occluder in an elderly patient with pneumothorax and subcutaneous emphysema by using a soft bronchoscope. The nickel-titanium alloy exposed by the VSD occluder is conducive to stimulating epithelialization or granulation tissue formation near the fistula, promoting the healing of the fistula, and reducing the risk of occluder displacement. Therefore, a VSD occluder can be selected for BPF diameters <8 mm.

*(3) PDA Occluder*. The PDA occluder is a mushroom-shaped device made of nitinol through a mesh weave, where the upper plate and waist are covered with a polyethyl ester film. Its placement requires a certain length of the stump to facilitate the fixation of the occluder. Fruchter et al. [48] treated five BPF patients using the AVP (PDA) technique, achieving a 100% success rate with no direct surgical complications recorded after a nine-month follow-up. One patient required two AVPs to seal two adjacent BPFs. The fistula diameters, however, were not mentioned in their study. Wang et al. [49] reported a successful one-time placement of a PDA occluder, under local anesthesia and flexible bronchoscopy guidance, for a BPF patient with an 8 mm fistula diameter. After implantation, bedside X-ray fluoroscopy showed that the occluder was fully released and in a good position. There were no complications, such as stent displacement, an irritating cough, or hemoptysis. Regular bronchoscopy re-examination showed that various degrees of granulation tissue hyperplasia appeared in the mucosa around the occluder, thereby wrapping the occluder, while there were no complications, such as local tissue necrosis around the fistula, fistula recurrence, occluder displacement, or local infection.

The article "Progress Report on Interventional Treatment for Bronchopleural Fistula" was published in 2023. Journal: Emerg Med Int.

However, the treatment specification for interventional therapy of BPF with an occluder has not yet been formed, and there are currently many disputes and doubts remaining [50]. Most occluder devices are still used beyond their specifications, and the original design cannot fully meet the requirements of the respiratory physiological environment. Therefore, large-scale studies and long-term follow-ups of clinical studies are still needed to confirm their safety and effectiveness.

#### 3.9.2. Linear Coils

Linear coils can be delivered through microcatheters, thereby allowing for the ultraselective occlusion of small structures, which are commonly used for arterial and venous embolization of peripheral vascular systems as well as aneurysms. Since these coils allow a high packing density, they offer a high probability of primary airtight occlusion and complete abolishment of air leakage. Guo et al. [51] used spring coil closure for the first time to treat a small fistula that had existed for up to 10 months in BPF patients. The tension formed by the spring ring in the tissue near the fistula was low, meaning that it was not easy to cause ischemia in the tissue close to the fistula, although the operation method is relatively simple and safe, and easy for patients. However, patients need to be followed up frequently to evaluate any complications such as an increased cough, infection, bleeding, or coil displacement. Baden et al. [52] reported the success of bronchoscopic superselective occlusion in a 1.2-year-old child with BPF using a removable high-density, large-capacity coil. The child was minimally traumatized, and long-term follow-up did not reveal any side effects or adverse events. Using coil plugging BPF, it is recommended to choose a small fistula with a diameter <5 mm and a certain fistula formation, which is conducive to the attachment of the spring ring and can reduce the risk of it falling off.

#### 3.9.3. Endobronchial Valve and Intrabronchial Valve

The endobronchial valve (EBV) was originally developed for lung volume reduction surgery in patients with severe emphysema. For relatively large bronchopleural fistulas, especially in patients with failed closure by medical adhesive, stents can stimulate granulation hyperplasia, promote fistula healing, and facilitate secretion drainage through a one-way valve function. Therefore, stents provide a safer and more effective means for the treatment of BPFs. Song et al. [53] reported that 26 patients received endobronchial valve placement, while the effective rate for BPF treatment was 73.1%. However, the common complications after endobronchial valve placement can include lung infection, granulation tissue formation, valve displacement, or prolapse. To reduce the risk of complications, EBV should be removed within 6 weeks of implantation, when the patient's condition stabilizes and their clinical symptoms disappear. Cheng et al. [54] used an EBV to treat two patients with BPF and achieved good results. They believed that an EBV could be attempted for 4–8 mm fistulas. This is similar to the research results of Song et al. [53]. Moreover, EBV-TS-4.0 can be selected for 4.0–6.5 mm fistulas, and EBV-TS-5.5 can be selected for 6.5–8.0 mm fistulas. If the fistulas are funnel-shaped, an endobronchial valve can be tried for occlusion. If the fistulas are located on the side wall rather than the blind end, the EBV may not be fixed and suitable for placement.

The article "Progress Report on Interventional Treatment for Bronchopleural Fistula" was published in 2023. Journal: Emerg Med Int.

The intrabronchial valve (IBV) is a small, umbrella-shaped apparatus designed to inhibit airflow toward the lung's distal end [55]. A flexible bronchoscopy facilitates its placement into the necessary airway and also its subsequent removal. Potential complications of IBV insertion include atelectasis, airway or tissue damage, distal infection, localized airway swelling or edema at the implantation site, persistent cough, hemoptysis, valve displacement, pneumothorax, dyspnea, tissue hyperplasia, or granuloma death at the implant site. In the United States, the Spiration IBV system is approved for humanitarian device exemption, utilized for treating persistent air leakage in patients with postpulmonary parenchymal resection. Off-label applications include treatment of BPF/PAL following spontaneous emphysema, iatrogenic, and septic thoracic infections subsequent to routine treatment failure. The IBV is typically removed after an adequate healing duration, typically around six weeks. The employment of these valves shortens hospitalization and reduces the risk of hospital-related complications [56].

#### 3.9.4. Endobronchial Watanabe Spigot

In 1991, Japanese scholars reported for the first time that BPF can be occluded with self-made silicone plugs, and in 2003, it was transformed into endobronchial silicone plugs, which have good biocompatibility and are mainly used for blocking the target bronchial lumen to reduce or stop air leakage [57]. The EWS has the benefit of being minimally invasive, enabling easy insertion or removal under bronchoscopy, without specialized instruments. However, it does come with potential complications such as infection and EWS migration [58]. The EWS features surface studs to mitigate migration risks and can be safely inserted, even in patients with severe systemic diseases. EWS that are 5 or 6 mm are suitable for occluding subsegmental bronchi, while 7 mm EWS can occlude segmental bronchi [59]. Uchida et al. [60] used EWS for endobronchial embolization in patients with BPF and empyema after esophagectomy to prevent any air leakage. After endobronchial embolization, the thoracic drainage tube was removed, and no complications caused by the insertion of EWS were observed. Thus, medium and large EWS can be used to control air leakage. Date et al. [61] used the traction method to place an endobronchial Watanabe spigot (EWS) for the treatment of BPF, achieving certain results, overcoming the difficulties of traditional EWS placements, simplifying the procedure, and reducing recent complications. Furthermore, the guide wire is directly inserted into the BPF without worrying about selecting the incorrect bronchial tube. However, this method is only suitable for patients undergoing fenestration and thoracic drainage. The push and slide method [58] is a method of endoscopic bronchial occlusion using an endobronchial Watanabe spigot that facilitates occlusion of the target bronchus rapidly and accurately using a guidewire. Instead, the push and slide method was used in order to detect the fistulae. It may be a valid treatment option for empyema with multiple bronchopulmonary fistulae. In cases of postoperative peripheral BPF, if the target bronchus can be identified, the use of EWS and digital drainage systems (e.g., Thopaz) for peripheral BPF bronchial occlusion is an appropriate choice [62]. The occlusion technique involving a guide sheath (GS) and curette enables clear visual of EWS throughout the surgical process. This method facilitates quick EWS insertion within two minutes and can also be used to insert the upper lobe bronchus for placement [63]. The procedures and methods for EWS placement present significant research potential for the present and the future.

The article "Progress Report on Interventional Treatment for Bronchopleural Fistula" was published in 2023. Journal: Emerg Med Int.

#### 3.9.5. Development of Bronchial Occluders Using 3D Printing Imaging Technology

The use of 3D printing imaging technology has the advantages of personalization, accuracy, and remoteness and can clearly display the internal structure of tissues and organs. It is a new manufacturing technology in the medical field. According to a randomized controlled study by Xiao et al. [64], the application of 3D printing imaging technology to individually customized bronchial occluders has significant clinical efficacy in the treatment of BPF patients, which can significantly shorten the operation time and reduce the incidence of adverse events.

## 4. Discussion

Owing to the recent widespread development of endoscopic intervention, endoscopic treatment of BPF has gradually replaced surgery. Nevertheless, a dearth of large-scale, multicenter, randomized controlled studies exists, which precludes direct comparison of two or more interventional treatment methods. Moreover, there are currently no convincing clinical guidelines concerning the interventional treatment of BPF. The success rates of treatments vary, and an optimal treatment method for BPF is yet to be universally acknowledged. Given the absence of standardized treatment recommendations, individual treatment strategies must be formulated taking into account the location of the bronchopleural or tracheal pleural fistula and any existing complications. Treatment selection may also be influenced by factors such as the size and location of the fistula, differing medical conditions, policies, and standards across various countries and regions, as well as the patient's economic status, comprehension, and acceptance of the treatment, and presence of other complications. Bronchoscopy intervention is the preferred initial choice for small BPFs with a diameter of less than 5 mm. Endoscopic closure of BPF is advantageous due to its lower cost, reduced incidence of trauma, and feasibility in critically ill patients. The author posits that, for patients with BPFs of a diameter less than 5 mm—particularly ≤ 3 mm sealing agents, hardening agents, or chemicals can all produce favorable therapeutic outcomes. For BPFs with a diameter greater than 5 mm, endobronchial nasal broncholavage (ENBL) has demonstrated efficacy. Airway stents, biomaterials, and occlusive devices are viable options for BPFs with a diameter of 8 mm or less. For BPFs of approximately 10 cm in diameter, treatment methods such as the application of ASD occluder and autologous fat have shown promising results. However, additional studies with larger samples are needed to assess their short-term and long-term efficacy and complications and refine their indications and contraindications. The future research focus will be on novel methods and equipment for BPF interventional treatment, including custom-made stents and occluders created with 3D printing technology, biological and chemical materials with superior treatment effects and fewer complications, and the complementary advantages of different treatment methods. These research outcomes will, to some degree, shape clinical practice, and the effectiveness of enhanced clinical practice will continue to enrich these research findings. Therefore, the ongoing advancements in interventional medicine and devices will prove beneficial for more patients afflicted with BPF.
